The article "KGF-2 Protects against Lung Ischemia-Reperfusion Injury by Inhibiting Inflammation-Induced Damage to Endothelial Barrier Function" was retracted in 2023. Reasons: signs of a paper mill; compromised peer review; unreliable results or conclusions.

# KGF-2 Protects against Lung Ischemia-Reperfusion Injury by Inhibiting Inflammation-Induced Damage to Endothelial Barrier Function

**DOI:** 10.1155/2022/3055039

**Published:** 2022-05-11

**Authors:** Fangfang Xia, Zhousheng Jin, Jiaojiao Dong, Chaoxing Chen, Yaoyao Cai, Quanguang Wang, Hongfei Chen

**Affiliations:** Department of Anesthesiology, The First Affiliated Hospital of Wenzhou Medical University, Zhejiang, Wenzhou, China

## Abstract

Lung ischemia-reperfusion injury (LIRI), which has a mortality rate of approximately 50%, is a popular topic in critical care research. Keratinocyte growth factor-2 (KGF-2) is secreted by mesenchymal cells, and it is effective in promoting the proliferation, migration, and differentiation of various epithelial cells. To date, however, only a few reports on KGF-2-related regulators in LIRI have been published. In the current study, an LIRI rat model is constructed, and the upregulation of the fibroblast growth factor receptor 2 (FGFR2) is observed in the LIRI rat model. In addition, LIRI induces NLRP1 inflammasome activation in vivo and in vitro, and KGF-2 inhibits LIRI-induced damage to pulmonary microvascular endothelial cells. Mechanistically, KGF-2 inhibits NLRP1 inflammasome and NF-*κ*B activity. KGF-2 inhibition attenuates LIRI injury-induced damage to endothelial integrity. In conclusion, KGF-2 protects against LIRI by inhibiting inflammation-induced endothelial barrier damage.

## 1. Introduction

Lung ischemia-reperfusion injury (LIRI) can occur due to trauma, atherosclerosis, pulmonary embolism, thrombosis, and some surgical procedures, such as cardiopulmonary bypass and lung transplantation [1]. LIRI has a certain incidence rate that can lead to serious clinical concurrence [2]. Inflammatory factors are activated during the early stage of LIRI; gas exchange becomes abnormal and lung compliance is reduced due to the dysfunction of the vascular endothelium and the alveolar epithelium [3]. The functional recovery of alveolar epithelial and endothelial cells is an important influencing factor in the recovery of patients with acute lung injury and respiratory distress [4]. To date, the research mechanism of LIRI remains unclear, although some related studies have been conducted. Through the in-depth study of ischemia-reperfusion injury in recent years, the activation of leukocytes and the injury of endothelial cells have been determined to play important roles. In the pathophysiological process of ischemia reperfusion, various inducing factors, inflammatory mediators, effector cells, and effectors form a complex network, and the “focus” of this network is NF-*κ*B. The transcription products regulated by NF-*κ*B are the primary inflammatory mediators and cytokines in the inflammatory response of ischemia-reperfusion injury, mostly including pre-inflammatory cytokines, such as tumor necrosis factor (TNF)-*α*, interleukin (IL)-1, IL-6, and IL-8, along with inflammatory mediators and adhesion molecules that aggregate leukocytes. Therefore, NF-*κ*B can regulate inflammation upstream, and it is the “hub” of inflammatory regulation in ischemia-reperfusion injury [5, 6]. Alternatively, several studies have suggested that p38 mitogen-activated protein kinase (MAPK) plays an important role in the development of LIRI by mediating lung endothelial cell barrier dysfunction. However, the mechanism of LIRI requires further research.

In 1996, keratinocyte growth factor-2 (KGF-2), which belongs to the family of fibroblast growth factors, was determined to be expressed primarily in the lungs [7]. The KGF-2 signaling pathway controls the survival and proliferation of endogenous distal alveolar progenitor cells through fibroblast growth factor receptor 2 (FGFR2)-IIIb, which is crucial for lung development [8]. At present, KGF-2 has been demonstrated to possibly inhibit DNA damage, apoptosis, and induced pulmonary fibrosis in epithelial cells, suggesting that KGF-2 may be a novel treatment for alveolar epithelial injury [9, 10]. KGF-2 was also found to increase angiogenesis [11]. Huisuo Hong et al. found that dexmedetomidine preconditioning ameliorates lung injury induced by pulmonary ischemia/reperfusion by upregulating promoter histone H3K4me3 modification of KGF-2 [12]. And research shows that keratinocyte growth factor-2 reduces inflammatory response to acute lung injury induced by oleic acid in rats by regulating key proteins of the Wnt/*β*-catenin signaling pathway [13].

However, the relationship between KGF-2 and lung injury and the function of endothelial cells during lung injury remain unclear. The objective of the current research is further to study the role and mechanism of KGF-2 in lung injury.

## 2. Materials and Methods

### 2.1. Construction of LIRI Rat Models

A total of 30 male Sprague–Dawley (SD) rats were randomly divided into three groups: the blank control, sham, and LIRI groups. The SD rats in the blank control group did not receive any treatment. The establishment of an LIRI model was described previously [13]. The operation process of the LIRI group was as follows: The rats were anesthetized through an intraperitoneal injection of pentobarbital sodium at 50 mg/kg and an intramuscular injection of atropine at 0.2 mg/kg. After disinfecting the skin of the neck with iodophor, the subcutaneous tissue and muscle were dissected and separated, and the trachea was exposed with a *T*-shaped incision. After cannulation, the rats were mechanically ventilated (Model 7025; Ugo Basile, Varese, Italy) with a standardized inspiratory oxygen fraction of 60% at a rate of 75 breaths/min, a tidal volume of 10 mL/kg, a positive end-expiratory pressure of 2 cm H_2_O, and an arterial partial pressure of CO_2_ at 30–45 mmHg. The skin was cut in the fifth intercostal space of a rat's left chest, and part of the muscle tissue was removed to expose the ribs. Subsequently, three, four, and five ribs were cut, the left thoracic cavity was opened, and the lung tissue was pulled with forceps. All the animals received 50 U of intravenous heparin. The pulmonary hilum, including the left main bronchus, artery, and vein, was occluded with a noncrushing microvascular clamp for 90 min. After the 90-min left lung ischemia, the clamp was removed and the lung was ventilated and reperfused for 4 h. The entire procedure must be gentle to avoid damaging the lung tissue. The operation of the sham group was the same as that of the LIRI group, except that the pulmonary hilum was not occluded. At the end of the reperfusion period, the partial pressure of oxygen (pO_2_) value was compared with the pre-ischemia value among different groups. At the end of the experiment, the lung tissue was collected for other trials.

In addition, 40 rats were randomly divided into 4 groups. The first group was treated with dimethyl sulfoxide (DMSO), while the second group was treated with KGF-2 (A single dose of KGF-2 (0.5 mg/kg) was injected intraperitoneally.). The third group was pretreated with DMSO before LIRI. The rats in the fourth group were pretreated with KGF-2 before LIRI (A single dose of KGF-2 (0.5 mg/kg) was injected intraperitoneally before operation.).

This study was approved by Ethics committee of the First Affiliated Hospital of Wenzhou Medical University (WMU-FY-071).

### 2.2. Culture of Rat Pulmonary Microvascular Endothelial Cells (rPMVECs)

Rat PMVECs (r PMVECs) were placed in a hypoxic incubator containing 95% N_2_ and 5% CO_2_ for 12 h under hypoxic conditions. Next, the culture medium was replaced with DMEM containing glucose, 1% penicillin-streptomycin, 10% FBS, and 4 mM L-glutamine for 4 h to construct the LIRI cell model. The cells were collected for subsequent experiments. For the LIRI + KGF-2, 20 mM KGF-2 (Libang Sciences) was added prior to the establishment of the LIRI cell model. NLRP1 overexpression plasmid (pcDNA3.1-NLRP1) and pcDNA3.1 NC were synthesized by Guangzhou RiboBio Co., Ltd. (Guangzhou, Guangdong, China). Transfection was performed using Lipofectamine® 3000 (50 nM; Thermo Fisher Scientific, Inc.) according to the manufacturer's protocol.

### 2.3. Hematoxylin and Eosin (HE) Staining Experiments

First, the lung tissue soaked in formalin was taken out. The tissue was trimmed, placed in an embedding box, and rinsed with running water for approximately 6 h. The tissue was placed in a dehydrator for 12 h to complete dehydration, and then it was taken out and embedded into paraffin. After the paraffin had completely solidified, tissue sections were prepared and dried at 60°C for 2 h. The dried tissue was first stripped of paraffin by using xylene and then treated with different concentrations of alcohol. Finally, the tissue was treated in distilled water. After dyeing with HE stain, the tissue was dehydrated in alcohol, made transparent by using xylene, and sealed with neutral gum. Finally, the morphological changes of the lung tissue were observed under a LEICA camera microscope (Wetzlar, Germany).

### 2.4. Immunohistochemical Experiment

The lung tissue stored in formalin was taken out. The tissue was trimmed, placed in an embedding box, and then rinsed with running water for approximately 6 h to remove the formalin. The tissue was then placed in a dehydrator for overnight dehydration, taken out of the embedding box, and embedded into paraffin. After the paraffin had completely solidified, the tissue was divided into sections. The tissue sections were placed on glass slides and dried at approximately 60°C for 3 h. Thereafter, the tissue was dewaxed and hydrated, and antigen repair was performed in a microwave oven. After the aforementioned solution had cooled naturally, the excess repair solution was cleaned with phosphate-buffered saline (PBS). The tissue was treated with goat serum that contained 10%, and the blocking solution was removed. Then, the corresponding primary antibodies were added, and the tissue was incubated overnight at 4°C. After cleaning the excess primary antibody with PBS, horseradish peroxidase-labeled secondary antibody was added, and the tissue was incubated in the dark at 37°C for 2 h. After cleaning the excess secondary antibody with PBS, 3,3′-diaminobenzidine (DAB) was added, and the staining was observed under a microscope. After dyeing, excess DAB was cleaned with PBS. After the tissue was treated with hematoxylin for 5–10 min, the excess hematoxylin was cleaned with PBS, and then the tissue was dehydrated and sealed. The staining of the tissue was observed under a LEICA camera microscope (Wetzlar, Germany) and recorded.

### 2.5. Detection of the Wet/Dry Weight Ratio of Lung Tissues

The rats were sacrificed, and their lung tissues were isolated. Water from the surface of the lung tissues was drained. Some parts of the lung tissues were kept for other tests, while the remaining parts were weighed. The lung tissues were placed in a 60°C oven for 72 h to obtain a constant weight and then weighed again. The net weight ratio of both lung tissues was the wet/dry weight ratio, which can reflect the degree of pulmonary edema or extravascular pulmonary edema.

### 2.6. Detection of the Total Protein Level in the Bronchoalveolar Lavage Fluid (BALF)

#### 2.6.1. Acquisition of BALF

After the rats were sacrificed, their lung tissues and main bronchi were removed. A rinse tube was inserted and fixed into the main bronchus before injecting 1.5 mL of PBS into the bronchus and then extracting it. After repeating the preceding steps three times, three washes were collected for total protein determination.

#### 2.6.2. Total Protein Extraction of Lung Tissues

Total protein extracts were added to 100 mg of lung tissue, and the homogenates were prepared. The supernatant was collected after centrifugation for 10 min at 10,000 rpm. Then, the total protein content was determined by following the procedure recommended by the total protein extraction kit (SD-001/SN-002; Invent BIOTECHNOLOGIES, INC, USA).

### 2.7. Enzyme-Linked Immunosorbent Assay (ELISA)

IL-8 (SEKR-0071; Solarbio, Beijing, China), IL-6 (ab234570; Abcam, MA, USA), IL-4 (ab100770; Abcam, MA, USA), IL-10 (ab214566; Abcam, MA, USA), and TNF-*α* (ab236712; Abcam, MA, USA) in peripheral venous blood and BALF were measured using ELISA kits in accordance with the manufacturer's instructions. The levels of cytokines IL-1*β* (ab255730; Abcam, MA, USA) in the supernatants of rPMVECs were also tested.

### 2.8. Real-Time Polymerase Chain Reaction (PCR) Test

Lung tissues or rPMVECs were placed on ice, and TRIzol was added and gently mixed for 5 min. Then, chloroform was added and the solution was mixed for 2–3 min. Thereafter, the solution was placed in a low-temperature centrifuge and centrifuged at 12,000 rpm for 15 min at 4°C. The supernatant was collected. After adding isopropanol, the supernatant was treated on ice for 4 min. Then, it was centrifuged for 10 min at 12,000 rpm at 4°C. After centrifugation, the supernatant was poured out, added with 75% alcohol, shaken gently, and placed in a low-temperature centrifuge for centrifugation at 4°C at 12,000 rpm for 5 min. Finally, the supernatant was removed and dissolved with enzyme-free water, determining the RNA concentration.

RNA was predenatured at 94°C for 5 min, followed by denaturation at 94°C for 30 s, annealing for 40 s at 57°C, and extension for 50 s at 72°C, for a total of 30 cycles. The final cycle had a temperature of 72°C and was extended for 10 min. Then, the content of related messenger RNA (mRNA) was measured. Refer to Table 1 for the specific sequence.

### 2.9. Terminal Deoxynucleotidyl Transferase (TdT) dUTP Nick End Labeling (TUNEL) Assay

Paraffin-embedded lung tissues were sectioned, dewaxed, and hydrated. Proteinase K solution was added at room temperature for 15 min to remove tissue proteins. Then, PBS with 2% hydrogen peroxide was added to the lung tissue sections for 5 min at room temperature. Subsequently, two drops of TdT enzyme buffer were added to the lung tissue sections for 1–5 min at room temperature. Next, TdT enzyme reaction solution was added dropwise to the slices and allowed to react at 37°C for 1 h. Then, washing and termination reaction buffer preheated to 37°C was added and maintained at 37°C for 30 min. Thereafter, peroxidase-labeled antibody was dropped to the slices and allowed to react for 30 min at room temperature. Finally, the sections were treated with DAB solution for 3–6 min and restained with methyl green for 10 min. The tissues were then dehydrated, sealed, and photographed under a LEICA camera microscope (Wetzlar, Germany).

### 2.10. Western Blot Analysis

The lung tissue was clipped and prepared into tissue homogenate, and a mixture of radioimmunoprecipitation assay buffer and phenylmethylsulfonyl fluoride was added to it. The lung tissue was placed in a cryogenic centrifuge and centrifuged for 15 min at 12,000 r/min at 4°C. After centrifugation, the supernatant was collected, and the protein concentration was determined.

Then, polyacrylamide gel electrophoresis was used to separate proteins with different molecular weights and transfer them to the nitrocellulose membrane. The nitrocellulose membrane was treated with 5% bovine serum albumin at room temperature for 1 h to block nonspecific binding sites. Then, different monoclonal antibodies were used to react with proteins on the nitrocellulose membrane at 4°C for 12 h. Subsequently, after washing the excess primary antibodies with a buffer solution, horseradish peroxidase-labeled secondary antibodies were incubated with the aforementioned nitrocellulose membrane for 2 h at room temperature. The contents of different proteins were then measured via X-ray diffraction.

### 2.11. Statistical Analysis

All data were presented as mean ± standard deviation. The statistical differences between groups were assessed via one-way ANOVA followed by Bonferroni correction. *P* < 0.05 indicated a statistically significant difference.

## 3. Results

### 3.1. Effect of Ischemia-Reperfusion Injury on Lung Tissue

After LIRI, the pO_2_, pathological morphology of lung tissues and apoptosis degree of lung epithelial cells were changed. Compared with those in the blank and sham groups, the value of pO_2_ in the LIRI group decreased significantly. However, no significant difference was observed between the sham and blank groups (Figure 1(a)). In the blank group, a small amount of inflammatory cell infiltration was seen in the lung stroma, and vascular congestion in the lung parenchyma was inevident. No obvious extravascular fluid retention occurred, the alveolar structure was clear, and no apparent fluid and cell exudation were noted. No significant difference was found between the sham and blank groups. In the LIRI group, however, interstitial lung tissue was thickened, and a large amount of inflammatory cell infiltration occurred. Blood vessels were congested in the lung interstitial, accompanied by hemorrhagic changes, exhibiting extravascular fluid retention, an unclear alveolar structure, large fluid and cell exudation in alveoli, and the formation of a hyaline membrane (Figure 1(b)). The results of the immunohistochemistry (IHC) and TUNEL assays showed no evident macrophage infiltration in the lung tissues and apoptosis of the lung epithelial cells in the blank and sham groups. In the LIRI group, however, a large amount of macrophage infiltration in the lung tissues and apoptosis of lung epithelial cells were observed (Figure 1(c) and 1(d)).

### 3.2. Upregulation of Inflammatory Factors and FGFR2 in the Lung Tissues of LIRI Rats

Figure 2(a) shows the effect of ischemia-reperfusion injury on the wet/dry weight ratio of lung tissues. The wet/dry weight ratio significantly increased in the LIRI group relative to the blank and sham groups, indicating a reduction in the consolidation formation of lung tissues and a significant increase in the water content of the LIRI group, suggesting significant pulmonary edema in the LIRI group. The results of the wet/dry weight ratio showed significant pulmonary edema in the LIRI group. We determined the expression of IL-6, IL-8, TNF-*α*, IL-4, and IL-10 inflammation-related factors in peripheral venous blood and BALF and used it to assess inflammatory response after LIRI. In Figure 2(b) and 2(c), the results showed that the expression of IL-6, IL-8, TNF-*α*, IL-4, and IL-10 was significantly increased in peripheral venous blood and BALF after LIRI, demonstrating that LIRI increased the rats' inflammatory response. In addition, we conducted PCR experiments to determine the content of FGFR2 mRNA in rat lung tissues after LIRI. The experimental results showed that the expression of FGFR2 mRNA increased after LIRI (Figure 2(d)). The aforementioned experimental results indicated that LIRI increased the expression of FGFR2 in lung tissues, resulting in pulmonary fibrosis.

### 3.3. LIRI Induces NLRP1 Inflammasome Activation In Vivo and In Vitro

As shown in Figure 3(a), we detected NLRP1 mRNA expression in rat lung tissues during the real-time PCR experiment. The results showed that NLRP1 mRNA expression in rat lung tissues increased significantly after LIRI. We performed Western blot assay to determine the expression of NLRP1, cleaved caspase-1, and cleaved-IL-1*β* in rat lung tissues. The result showed that the expression of NLRP1, cleaved caspase-1, and cleaved-IL-1*β* protein increased significantly in rat lung tissues after LIRI (Figure 3(b)). Moreover, we performed real-time PCR and Western blot assays to detect the mRNA motor neurone disease protein expression of NLRP1, cleaved caspase-l, and cleaved-IL-1*β* in rPMVECs after LIRI treatment. The result showed that the expression of NLRP1, cleaved caspase-1, and cleaved-IL-1*β* protein increased significantly in rPMVECs after LIRI (Figure 3(c) and 3(d)). The expression of IL-1*β* in LIRI-treated rPMVECs was further measured via ELISA. Consistent with the Western blot results, IL-1*β* expression increased in LIRI-treated rPMVECs (Figure 3(e)).

### 3.4. KGF-2 Suppresses LIRI-Induced rPMVEC Injury

The lung tissue morphology was similar in the DMSO and KGF-2 groups, and alveolar wall thickness and interstitial space were relatively normal, without evident infiltration of inflammatory cells and hemorrhage. Compared with the DMSO and KGF-2 groups, lung histopathology showed that lung tissues after LIRI and DMSO exhibited a significant increase in the thickness of the alveolar wall and interstitial space, the number of infiltrating leukocytes in the lung tissues and alveolar space, and plasma exudation within the alveoli. Some red blood cells were found in the interstitial tissue and alveolar space. Several alveoli became larger, and they were either filled with liquid or had collapsed. The changes in lung tissue morphology in LIRI rats treated with KGF-2 were alleviated. The lung injury score can determine lung injury severity. The results showed that the severity of lung injury in the LIRI group was significantly higher than those in the DMSO and KGF-2 pretreatment groups (Figure 4(a)). The wet/dry weight ratio of lung tissues reflects the degree of pulmonary edema. The wet/dry weight ratios of the lung tissues of the DMSO and KGF-2 groups were lower, but the wet/dry weight ratio of lung tissues after LIRI and DMSO treatment increased significantly, indicating that the degree of pulmonary edema was more serious. However, the wet/dry weight ratio of lung tissues in the LIRI group pretreated with KGF-2 decreased and alleviated pulmonary edema (Figure 4(b)). The total protein level in BALF of the DMSO and KGF-2 groups was lower, and no significant difference was observed between them. The total protein level in the BALF of rats co-treated with LIRI and DMSO increased significantly. Although the total protein level in the BALF of LIRI rats pretreated with KGF-2 was still higher than that of rats treated only with DMSO and KGF-2, it was considerably lower than that of rats co-treated with LIRI and DMSO. This result showed that the permeability of pulmonary endothelial cells increased (Figure 4(c)).

### 3.5. KGF-2 Inhibition Attenuates LIRI Injury-Induced Damage to Endothelial Integrity

Protein expression levels, such as those of aquaporin I (AQP1), intercellular adhesion molecule I (CAM-1), zonulae occludente 1 (ZO-1), vascular endothelial cadherin (VE-cadherin), phosphorus (P)-p38 MAPK, and p38 MAPK, in lung tissues can explain the integrity of endothelial cells. To confirm that KGF-2 pretreatment can alleviate the change in P-p38 MAPK, p38 MAPK, AQP1, ICAM-1, ZQ-1, and VE-cadherin caused by LIRI and the destruction of the endothelial barrier, we performed Western blot to observe the expression of P-p38 MAPK, p38 MAPK, AQP1, ICAM-1, ZO-1, and VE-cadherin in the lung tissues of each group. The results showed a slight difference in the expression of p38 MAPK, AQP1, ICAM-1, ZO-1, and VE-cadherin in the lung tissues of rats treated only with DMSO and KGF-2. After LIRI treatment, however, the expression of p38 MAPK and ICAM-1 increased significantly, while those of AQP1, ZO-1, and VE-cadherin were significantly decreased in rat lung tissues. Although the expression of p38 MAPK and ICAM-1 in rat lung tissues in the KGF-2 pretreatment group still increased and the expression of AQP1, ZO-1, and VE-cadherin still decreased compared with those in the group treated only with DMSO and KGF-2, the expression of p38 MAPK und ICAM-I was significantly decreased and that of AQP1, ZO-1, and VE-cadherin was significantly increased compared with those in the LIRI group (Figures 5(a)–5(f)).

### 3.6. KGF-2 Inhibits NLRP1 Inflammasome and NF-*κ*B Activity

To demonstrate that KGF-2 is associated with NLRP1 and NF-*κ*B, we conducted a Western blot experiment to verify NLRP1 and cleaved caspase-1 expression in different groups. Compared with the protein expression of NLRP1and cleaved caspase-1 in the LIRI group, the expression of NLRP1 and cleaved caspase-1 was significantly decreased in rPMVECs pretreated with KGF-2 before LIRI. Meanwhile, the expression of NLRP1 and cleaved caspase-l in rPMVECs transfected with pcDNA3.1-NLRP1 increased but was still lower than that in the LIRI group (Figures 6(a) and 6(b)). We collected the medium from rPMVECs and performed ELISA to detect IL-1*β* in the medium. The results showed that the expression of IL-1*β* in the KGF-2 pretreatment group before rat LIRI was the least, the expression of IL-1*β* in the LIRI group was the highest, and the expression of IL-1*β* transfected with NLRP1 was in between the two (Figure 6(c)). Furthermore, we verified the protein levels of p-p65 and I*κ*B via Western blot. The results showed that, compared with those in the sham group, the level of p-p65 protein increased significantly and the level of I*κ*B protein decreased significantly in the LIRI group. When treated with KGF-2, however, the preceding situation was alleviated. That is, the expression of p-p65 protein was reduced and that of I*κ*B was increased. However, the p-p65 protein level was the highest and the I*κ*B protein level was the lowest in the LIRI group (Figures 6(d) and 6(e)).

## 4. Discussion

LIRI is considered a serious complication that can lead to a high incidence rate and mortality. LIRI mostly occurs during lung transplantation or cardiopulmonary bypass. It is one of the greatest challenges in postoperative nursing. LIRI can lead to acute lung injury and even more serious fatal complications, such as adult respiratory distress syndrome [14]. In recent years, many mechanisms, such as oxidative stress, aseptic immunity, complement activation, activation of coagulation pathway, endothelial dysfunction, and apoptosis [15], have been considered the pathogenesis of ischemia-reperfusion injury [16, 17]. The mechanisms of LIRI are complex and overlapping, but clarifying them can help prevent potentially serious complications. KGF-2 is primarily expressed in the lungs [18], but it is also widely expressed in other tissues; it is involved in angiogenesis, mitosis, cell differentiation, and migration [19–21]. KGF can induce minor angiogenesis and maintain the barrier function in the capillary monolayer. Given that the structure of KGF-2 is similar to that of KGF, we can predict that KGF-2 should have a similar function in blood vessels [11, 18]. At present, a small number of studies on the relationship of KGF-2 to lung ischemia and perfusion have been conducted; however, research on the pathway or mechanism by which KGF-2 affects LIRI and rPMVEC injury remains lacking. The objective of the current work is to study the role of KGF-2 in LIRI and the pathway through which KGF-2 plays its role.

We investigated the decrease in pO_2_ in the rat pulmonary vein after LIRI by establishing an LIRI rat model. Moreover, we confirmed through HE staining and IHC and TUNEL assays that lung tissue morphology changed after LIRI. These changes included thickened interstitial lung tissues, a large number of inflammatory and macrophage cell infiltration, congested blood vessels in the lung interstitial, hemorrhagic changes, extravascular fluid retention, unclear alveolar structure, large fluid and cell exudation in alveoli, and the apoptosis of lung epithelial cells. We further investigated the wet/dry weight ratio of rat lung tissues after LIRI, demonstrating that rat lung edema occurred after LIRI. In addition, we examined the expression of associated inflammatory factors, such as IL-6, IL-8, TNF-*α*, IL-4, and IL-10, in peripheral venous blood and BALF after LIRI. The results of which indicated that LIRI caused an inflammatory response. The expression of FGFR2 in lung tissues was further confirmed to increase significantly after LIRI, inducing pulmonary fibrosis. Our experimental results also showed a certain relationship between LIRI and NLRP1 inflammasome activation. We determined that the protein and mRNA levels of NLRP1 inflammasome, cleaved caspase-l, and cleaved IL-1*β* in rat lung tissues and rPMVECs increased significantly after LIRI. Moreover, the expression of IL-1*β* in rPMVECs also increased significantly. The preceding experimental results clearly showed that LIRI can induce lung tissue and rPMVEC inflammatory response. The role played by KGF-2 in LIRI is the focus of our study. The experimental results confirmed that KGF-2 can alleviate LIRI-induced changes in lung tissue morphology and relieve LIRI-induced pulmonary edema and lung tissue permeability. For example, KGF-2 pretreatment can reduce the wet/dry weight ratio of lung tissues after LIRI, i.e., alleviate pulmonary edema. KGF-2 pretreatment can improve the total protein level in BALF after LIRI, indicating that KGF-2 can reduce the changes in lung permeability caused by LIRI. That is, KGF-2 can alleviate LIRI-induced lung and rPMVEC injuries. LIRI can change lung permeability, indicating that pulmonary endothelial cells may be damaged. We further studied the effect of KGF-2 on the integrity of pulmonary endothelial cells after LIRI. By detecting proteins' levels related to endothelial integrity, we proved that KGF-2 can effectively reduce the levels of p38 MAPK and ICAM-I proteins and increase the levels of AQP1 ZO-1 and VE-cadherin proteins. That is, KGF-2 inhibition attenuates LIRI injury-induced damage to endothelial integrity. Finally, we studied the relationship of KGF-2 to NLRP1 inflammasome and NF-*κ*B. The experimental results showed that KGF-2 can effectively reduce NLRP1 inflammasome, cleaved caspase-1, IL-1*β*, and p-p65, and enhance the expression of I*κ*B. This finding suggests that KGF-2 may play a role in protecting against lung and microvascular injuries by inhibiting the NLRP1 inflammasome and NF-*κ*B signaling pathways.

Our study confirmed that KGF-2 can alleviate lung injury caused by LIRI and may play a role in protecting against lung and microvascular injuries by inhibiting the NLRP1 inflammasome and NF-*κ*B signaling pathways. However, the specific mechanism of lung and microvascular injuries caused by LIRI should be further studied.

## Figures and Tables

**Figure 1:** Construction of LIRI rat models. (a) Graft pulmonary vena pO_2_ after LIRI. (b) Pathological changes in lung tissues after LIRI examined via HE staining (scale bar = 200 *μ*m). (c) Infiltration of macrophages (F4/80) in lung tissues after LIRI examined via IHC. (d) Apoptosis of pulmonary epithelial cells after LIRI examined via TUNEL assay (scale bar = 200 *μ*m). ^*∗*^*P* < 0.05 vs. control group. ^*∗∗*^*P* < 0.01 vs. sham group.

**Figure 2:** Upregulation of FGFR2 in LIRI rat models. (a) Wet/dry weight ratio of lung tissues after LIRI. (b) Expression of IL-6, IL-8, TNF-*α*, IL-4, and IL-10 in peripheral venous blood after LIRI. (c) Expression of IL-6, IL-8, TNF-*α*, IL-4, and IL-10 in BALF after LIRI. (d) Expression of FGFR2 in lung tissues after LIRI examined via real-time PCR. ^*∗*^*P* < 0.05, ^*∗∗*^*P* < 0.01 vs. sham group.

**Figure 3:** LIRI induces NLRP1 inflammasome activation in vivo and in vitro. (a) NLRP1 mRNA expression in rat lung tissues was detected via real-time PCR. (b) The protein levels of NLRP1, cleaved caspase-1, and cleaved-IL-1*β* were determined via Western blot in rat lung tissues. (c) Real-time PCR assay for the mRNA expression of NLRP1 in rPMVECs with or without LIRI treatment. (d) Western blot and densitometric analysis for the protein expression of NLRP1, cleaved caspase-1, and cleaved-IL-1*β* in rPMVECs. (e) Secretion of IL-1*β* in LIRI-treated rPMVECs measured via ELISA. *N* = 3; data are presented as mean ± SD; ^*∗*^*P* < 0.05, ^*∗∗*^*P* < 0.01, ^*∗∗∗*^*P* < 0.001 vs. sham group.

**Figure 4:** KGF-2 suppresses LIRI-induced rPMVEC injury. (a) Lung sections were stained with HE, and morphological changes were assessed. Magnification (scale bar = 200 *μ*m). (b) Wet/dry weight ratios of lung tissues as an index of lung edema. (c) Quantification of total protein in BALF. ^*∗*^*P* < 0.05.

**Figure 5:** KGF-2 inhibits NLRP1 inflammasome and NF-*κ*B activity. (a)–(f) Western blot of p-p38 MAPK, p38 MAPK, AQP1, ICAM-1, ZO-1, and VE-cadherin in lung tissues. Levels were normalized to that of the control, which was defined as 1.0. ^*∗*^*P* < 0.05, ^*∗∗*^*P* < 0.01, ^*∗∗∗*^*P* < 0.001.

**Figure 6:** KGF-2 inhibition attenuates LIRI injury-induced damage to endothelial integrity. (a) rPMVECs were transfected with or without pcDNA3.1-NLRP1 (NLRP1) plasmid for 24 h and then treated with 20 mM KGF-2 for 24 h before LIRI treatment. Western blot and densitometric analysis ((a) and (b)) of the protein levels of NLRP1 and cleaved caspase-1. (c) IL-1*β* levels in the culture media of rPMVECs were detected via ELISA. (d)–(e) Protein levels of p-p65 and I*κ*B were analyzed via Western blot. *N* = 3; data are presented as mean ± SD; ^*∗*^*P* < 0.05 vs. control group; ^#^*P* < 0.05 vs. LIRI group.

**Table 1:** Primer sequences.

Genes	Forward primer	Reversed primer
FGFR2	CCTGCGGAGACAGGTTTCG	TTGCCCAGCGTCAGCTTATC
NLRP1	TCCTATGAAGTAGTGCGGGC	TAACAGAGACCCCCACCTAAC

## Data Availability

The data used to support the findings of this study are available from the corresponding author upon request.
